RETRACTED

# SIRT2-KLF4 Interactions are Critical for Myeloma Survival and Migration

**DOI:** 10.1155/2022/7356477

**Published:** 2022-05-27

**Authors:** Chunjuan Lu, Jin Wei

**Affiliations:** ^1^Department of Blood Transfusion, Heilongjiang Provincial Hospital, Harbin, Heilongjiang 150036, China; ^2^Department of Nutrition, Heilongjiang Provincial Hospital, Harbin, Heilongjiang 150036, China

## Abstract

**Objective:**

To investigate the roles and possible mechanisms of SIRT2 and KLF4 in the development and progression of myeloma.

**Methods:**

Rt-PCR was used to detect SIRT2 in myeloma samples from patients and myeloma cells, the expression level of KLF4 in myeloma cells, and the effect of downregulation of SIRT2 expression on KLF4 expression level. MTT assay and wound-healing assay were used to observe the proliferation and migration of U266cells transient transfected with Sirt2 inhibitors.

**Results:**

SIRT2 is highly expressed in myeloma, but KLF4 was down. Downregulation of SIRT2 expression stimulated the expression level of KLF4. Reduced SIRT2 activity results in the release of KLF4 expression, which inhibits the proliferation and migration of myeloma cells.

**Conclusion:**

SIRT2-KLF4 combination plays an important role in the occurrence and development of myeloma.

## 1. Introduction

Myeloma is a malignancy associated with levels of monoclonal (M) protein in blood or serum and characterized by infiltration of malignant plasma cells in the bone marrow [1, 2]. Bone disease, hypercalcemia, renal insufficiency, cytopenia, and peripheral neuropathy are the main clinical manifestations of myeloma [3, 4]. The treatment of myeloma has made breakthrough progress in the fields of stem cell transplantation, targeted drug therapy, and homologous xenotransplantation [5, 6]. However, the high recurrence, heterogeneity, and other problems make it still a major intractable problem facing clinical medicine at present [7, 8].Therefore, the pathogenesis of myeloma at the molecular level needs to be investigated, and more accurate treatment methods need to be developed.

Sirtuin2 (SIRT2) is a member of the sirtuins family with NAD + dependent protein deacetylase activity [9, 10]. Previous studies have shown that SIRT2 is involved in many biological and pathological processes, such as cell movement and migration, microtubule dynamics, the development of leukemia, neurodegenerative disease, and the development of drug resistance [11–14]. In addition, abnormal expression of SIRT2 is related to the malignant progression of a variety of tumors, which can not only affect the progression of the tumor cell cycle but also change the tumor microenvironment [15, 16]. As a tumor suppressor gene, SIRT2 showed a low expression pattern in breast cancer and lung cancer tissues, which was different from that in normal tissues [14, 17]. On the contrary, in liver cancer and gastric cancer tissues, Sirt2 acts as an oncogene to promote tumor cell development and tumor metastasis [18, 19].

RETRACTED

The Kruppel-like factor 4 (KLF4), first isolated from the NIH3T3 cDNA library in 1994, is also known as GKLF [20, 21]. As a universal transcription factor, KLF4 exists in a wide range of organisms, from zebrafish to humans, and remains highly conserved [22]. Originally, KLF4 was identified as a gut-enriched factor that regulates the intestinal endoepithelial environment [23]. Subsequent studies have shown that KLF4 plays important roles in a variety of organs, such as improving corneal epithelial and skin barrier function [24, 25], coordinating bone cell differentiation [26], and promoting sperm vocalization [27]. The role of KLF4 in cancer development also has two sides [28]. On the one hand, KLF4 is usually lost in gastric, colorectal, and prostate cancers as a tumor suppressor gene [29]. On the contrary, KLF4 can also promote cancer development in an environmentally relevant way, such as primary ductal carcinoma of the breast [29].

These data suggest that SIRT2 and KLF4 are critical for tumor development, but their expression patterns and potential roles in myeloma remain unclear. The purpose of this study was to explore the important role of SIRT2 synergistically with KLF4 in myeloma survival and metastasis while exploring the expression of SIRT2 and KLF4 in myeloma.

## 2. Materials and Methods

### 2.1. Patients

Bone marrow samples were collected from 20 myeloma patients from December 2020 to September 2021 (age: 27–54; nine men and eleven women). All patients were adults (>18), had never received chemotherapy or radiation, and had no other hematologic malignancies or solid tumors. In addition, 8 healthy bone marrow samples were collected from 8 bone marrow donors as controls (age: 27 : 45; five men and three women). All procedures followed are carried out by the ethical standards of the Committee on Responsibility for Human Experimentation (Institutional and National) and following the 1975 Declaration of Helsinki, as amended in 2008.

### 2.2. Cell Culture

Myeloma cell lines KMS 28BM and U266 are preserved in our laboratory. Unless otherwise stated, all cells were cultured in RPMI-1640 medium supplemented with 15% FBS. Culture with 1% penicillin and streptomycin in a 5% CO_2_ humidified incubator is kept at 37°C.

### 2.3. RT-PCR

Total RNA was extracted from bone marrow samples or cells, and nucleic acid/protein analyzers and gel electrophoresis were used to determine the quality and quantity of RNA. Complementary DNA (cDNA) was obtained using the Thermo Scientific Kit. Bio-rad Minioption real-time PCR detection system and SYBR Green Super Mix were used for real-time quantitative PCR analysis. The gene expression level was analyzed by 2^−∆∆Ct^ method. Real-time PCR primer sequences are shown in Table 1.

RETRACTED

### 2.4. MTT Assay

Cell proliferation was determined by MTT assay. Cells in the logarithmic growth phase were collected according to the instructions and cell viability was determined at 24, 48, and 72 hours using CellTiter 96 AQueousOne Solution Cell Proliferation assay kit (Promega).

### 2.5. Wound-Healing Assay

The cells were routinely cultured overnight in six-well plates. The next day the pipette suction head was used to create artificial wounds at the bottom of each orifice plate. Cell migration and scratch healing were observed and photographed at 0 h and 24 h to quantify the degree of wound healing.

### 2.6. Statistical Analysis

All data were averaged after three experiments were repeated. Data were processed and statistically analyzed using Graphpad Prism 6.0. Statistical results were expressed as Mean ± SD, and *P* < 0.05 meant statistically significant differences. Photoshop CS6 was used for drawing and image processing.

## 3. Result

### 3.1. SIRT2 Is Upregulated in Myeloma Patients

To determine SIRT2 expression in myeloma samples, we used RT-QPCR to determine SIRT2 mRNA expression levels in 20 myeloma samples from patients and 8 normal bone marrow samples. The results showed that, as shown in Figure 1, SIRT2 mRNA expression was significantly increased in myeloma compared with normal tissues.

### 3.2. SIRT2 Is Upregulated in Myeloma Cells

Next, we measured SIRT2 mRNA expression in control cells and myeloma cells KMS 28BM and U266. Results, as shown in Figure 2, compared with the control group, the relative expression level of SIRT2 mRNA in KMS 28BM and U266cells was significantly increased.

In summary, the experimental data indicate that Sirt2 mRNA levels in both myeloma samples and myeloma cells show a high expression pattern different from that in normal tissues.

### 3.3. KLF4 Is Downregulated in Myeloma Cells

Considering the uncertainty and important role of KLF4 in tumor tissues, we first measured the expression of KLF4 mRNA in KMS 28BM and U266 myeloma cells and control cells. The results showed that the relative expression of KLF4 was significantly decreased in myeloma cells compared with control cells.  Figure 3 shows the expression of KLF4 in myeloma cells.

### 3.4. Inhibition of SIRT2 Reduce the Expression of KLF4

To investigate whether the expression changes of SIRT2 would affect the expression level of KLF4, we used SIRT2 inhibitors to instantaneously transfect myeloma cells U266 in the following experiments to inhibit the expression of endogenous SIRT2. Rt-qPCR confirmed that SIRT2 inhibitors reduced SIRT2 expression. Meanwhile, the expression level of KLF4 in myeloma cells with reduced SIRT2 expression was determined. The results showed that reduced SIRT2 expression in myeloma cells enhanced the KLF4 mRNA expression level.  Figure 4 shows expression of SIRT2 and KLF4 after transfection with SIRT2 inhibitor.

RETRACTED

### 3.5. Downregulated of SIRT2 and KLF4 Reduce Myeloma Cell Proliferation and Migration

In order to determine the effect of SIRT2 and KLF4 expression on U266 proliferation, an MTT assay was carried out next. The results showed that inhibition of SIRT2 expression resulted in a significant decrease in the proliferation rate of myeloma cells at 24 h compared with the control group (Figure 5). Scratch assay was used to evaluate the migration ability of myeloma cells after low expression of SIRT2. At 24 h, inhibition of SIRT2 expression also inhibited the migration ability of myeloma cells (Figure 6).

## 4. Discussion

Myeloma, a disease of the older population, is the second most common hematological malignancy [30]. In the past, new therapies such as immunomodulatory drugs and protease inhibitors have been developed in addition to autologous stem cell transplantation [31]. These treatments extend survival to some extent, but myeloma is still fundamentally incurable [32]. Therefore, it is very important to explore the genesis and development mechanism of myeloma from the genetic level.

The expression of transcription factors plays an important role in the occurrence and development of cancer, just as the high expression of IF1 affects the specificity of breast cancer migration and invasion [33]. According to previous reports, the expression and role of SIRT2 in myeloma are somewhat controversial. On the one hand, SIRT2 expression is reduced in myeloma patients, and its low concentration is associated with advanced disease and REDOX imbalance [34]. On the other hand, it has been reported that SIRT2 is highly expressed in myeloma patients [35]. To determine SIRT2 expression level in myeloma, we first collected samples from 20 myeloma patients and normal bone marrow samples from 8 volunteers. Rt-PCR results showed higher SIRT2 mRNA expression levels in myeloma patients compared with the control group. Subsequent experiments also verified this result, namely, the SIRT2 expression levels of myeloma cells KMS 28BM and U266 were significantly increased compared with control cells. These results indicated that SIRT2 showed a high expression pattern both in patients and in myeloma cells.

RETRACTED

KLF4 is a member of the Kruppel-like factor family and shows a high expression pattern in various tissues of the human body, such as differentiated and post-mitotic gastrointestinal epithelial cells. KLF4 is reported to be low expressed in tumor tissues as a tumor suppressor and has inhibitory effects on tumor cell proliferation and differentiation. The loss of KLF4 expression is often considered to be a predictor of poor survival. KLF4 plays a negative regulatory role in gastrointestinal tumors by interacting with TGF-*β*, Wnt/*β*-catenin, Notch, and other signaling pathways. KLF4 exerts its anticancer activity by inhibiting epithelial mesenchymal transformation of tumor cells [36]. This suggests that KLF4 is necessary for the maintenance of epithelial phenotypes in breast cancer cell MCF-10A epithelial cells. At the same time, KLF4 needs to maintain the expression of its downstream target E-cadherin to prevent the mesenchymal transformation of breast tumor epithelial cells, so as to play its role in inhibiting breast cancer metastasis [37]. In prostate cancer, epithelial mesenchymal transformation is involved in the progression of prostate cancer. KLF4 and FOXA1 directly inhibit SLUG expression in mouse and human prostate cancer cells. KLF4 acts as an inhibitor of Slug/Snail2 in prostate cancer cells [38]. However, the expression and role of KLF4 in myeloma have not been reported. In our study, KLF4 was found to have low expression of KMS 28BM and U266 in myeloma cells. It was also found that the KLF4 signal was released after SIRT2 expression was decreased in myeloma cells. This indicates that there is a potential relationship between SIRT2 and KLF4. The underlying mechanism of this association requires further study.

The strong proliferation and migration of tumors are key steps for their invasion to surrounding tissues and blood vessels so that they can develop into solid tumors through tumor angiogenesis and then metastasize to the distal site [39]. To prove the effects of SIRT2 and KLF4 on the proliferation and migration of myeloma cells, MTT analysis and scratch test were performed to detect the migration and proliferation of myeloma after transient transfection of SIRT2 inhibitor. The results showed that the proliferation and migration of myeloma cells were significantly inhibited after SIRT2 expression was decreased. KLF4 is reported to inhibit tumor angiogenesis [40]. In addition, it was proved in our experiment that KLF4 signal was significantly enhanced after downregulated SIRT2 expression. These results indicate that SIRT2 may inhibit KLF4 expression. When SIRT2 expression was weakened, KLF4 expression was released, which inhibited the proliferation and migration of myeloma cells.

RETRACTED

In summary, it was found in our study that SIRT2 was highly expressed in myeloma blood samples and myeloma cells, while KLF4 was less expressed in myeloma cells. Reduced SIRT2 activity releases KLF4 expression and inhibits myeloma cell proliferation and migration. SIRT2 and KLF4 are expected to be emerging therapeutic targets for myeloma.

## Figures and Tables

**Figure 1:** The expression of SIRT2 in myeloma patients.

**Figure 2:** The expression of SIRT2 in myeloma cells.

**Figure 3:** The expression of KLF4 in myeloma cells.

**Figure 4:** Expression of SIRT2 and KLF4 after transfection with SIRT2 Inhibitor.

**Figure 5:** The cell viability at various time points following transfection.

**Figure 6:** The Cell healing rate at various time points following transfection.

**Table 1:** Oligonucleotide primers used in RT-PCR studies.

Gene	Forward primer	Reverse primer
GAPDH	GAAGGTGAAGGTCGGAGTC	GAAGATGGTGATGGGATT TC
SIRT2	ACGCTGTCGCAGAGTCAT	CGCTCCAGGGTATCTATGTT
KLF4	TCCCGACCAGAGAGAACGAACG	ACAATCAGCAAGGCGAGTAAGTAGG

## Data Availability

No data were used to support the findings of the study.

## References

[1] Hideshima T., Mitsiades C., Tonon G., Richardson P. G., Anderson K. C. (2007). Understanding multiple myeloma pathogenesis in the bone marrow to identify new therapeutic targets. *Nature Reviews Cancer*.

[2] van de Donk N. W. C. J., Pawlyn C., Yong K. L. (2021). Multiple myeloma. *The Lancet*.

[3] Kumar S. K., Rajkumar V., Kyle R. A. (2017). Multiple myeloma. *Nature Reviews Disease Primers*.

[4] Kazandjian D. (2016). Multiple myeloma epidemiology and survival: a unique malignancy. *Seminars in Oncology*.

[5] Gertz M. A., Ansell S. M., Dingli D. (2008). Autologous stem cell transplant in 716 patients with multiple myeloma: low treatment-related mortality, feasibility of outpatient transplant, and effect of a multidisciplinary quality initiative. *Mayo Clinic Proceedings*.

[6] Fermand J. P., Ravaud P., Chevret S. (1998). High-dose therapy and autologous peripheral blood stem cell transplantation in multiple myeloma: up-front or rescue treatment? Results of a multicenter sequential randomized clinical trial. *Blood*.

[7] Mattia D. A, Marco S, Antonio P, Alessandra L, Francesca G (2017). Novel investigational drugs active as single agents in multiple myeloma. *Expert Opinion on Investigational Drugs*.

[8] Zhao W.-H., Liu J., Wang B.-Y. (2018). Updated analysis of a phase 1, open-label study of LCAR-B38M, a chimeric antigen receptor T cell therapy directed against B-cell maturation antigen, in patients with relapsed/refractory multiple myeloma. *Blood*.

RETRACTED

[9] Swyter S., Schiedel M., Monaldi D. (2018). New chemical tools for probing activity and inhibition of the NAD + -dependent lysine deacylase sirtuin 2. *Philosophical Transactions of the Royal Society B: Biological Sciences*.

[10] Youm Y.-H., Nguyen K. Y., Grant R. W. (2015). The ketone metabolite *β*-hydroxybutyrate blocks NLRP3 inflammasome-mediated inflammatory disease. *Nature Medicine*.

[11] Liu G., Park S.-H., Imbesi M. (2017). Loss of NAD-dependent protein deacetylase sirtuin-2 alters mitochondrial protein acetylation and dysregulates mitophagy. *Antioxidants and Redox Signaling*.

[12] Patel V. P., Chu C. T. (2014). Decreased SIRT2 activity leads to altered microtubule dynamics in oxidatively-stressed neuronal cells: implications for Parkinson’s disease. *Experimental Neurology*.

[13] Taylor D., Pallos J., Lambert E. (2010). A10 SIRT2 inhibition achieves neuroprotection by decreasing sterol biosynthesis. *Journal of Neurology, Neurosurgery & Psychiatry*.

[14] Kosuke F., Tomoatsu H., Kanae E. (2018). SIRT2‐mediated inactivation of p73 is required for glioblastoma tumorigenicity. *EMBO Reports*.

[15] Tang Y., He Y., Zhao N., Chen Y., Xing J., Tang N. (2022). Sirtuin2 correlates with lymph node metastasis, increased FIGO stage, worse overall survival, and reduced chemosensitivity to cisplatin and paclitaxel in endometrial cancer. *Irish Journal of Medical Science*.

[16] Zhang L., Kim S., Ren X. (2020). The clinical significance of SIRT2 in malignancies: a tumor suppressor or an oncogene?. *Frontiers Oncology*.

[17] Fiskus W., Coothankandaswamy V., Chen J. (2016). SIRT2 Deacetylates and Inhibits the Peroxidase Activity of Peroxiredoxin-1 to Sensitize Breast Cancer Cells to Oxidant Stress-Inducing Agents. *Cancer Research*.

[18] Chen J., Chan A. W. H., To K.-F. (2013). SIRT2 overexpression in hepatocellular carcinoma mediates epithelial to mesenchymal transition by protein kinase B/glycogen synthase kinase-3*β*/*β*-catenin signaling. *Hepatology*.

[19] Yang L., Zhang M., Dorfman R. G. (2018). SIRT2 promotes the migration and invasion of gastric cancer through RAS/ERK/JNK/MMP-9 pathway by increasing PEPCK1-related metabolism 1 2. *Neoplasia*.

[20] Shields J. M., Christy R. J., Yang V. W. (1996). Identification and characterization of a gene encoding a gut-enriched krüppel-like factor expressed during growth arrest. *Journal of Biological Chemistry*.

[21] Xiang F., Zhu Z., Zhang M. (2021). 3,3’-Diindolylmethane enhances paclitaxel sensitivity by suppressing DNMT1-mediated KLF4 methylation in breast cancer. *Frontiers Oncology*.

[22] Morales-Martinez M., Vega G. G., Neri N. (2020). MicroRNA-7 regulates migration and chemoresistance in non-hodgkin lymphoma cells through regulation of KLF4 and YY1. *Frontiers Oncology*.

RETRACTED

[23] Ghaleb A. M., McConnell B. B., Kaestner K. H., Yang V. W. (2011). Altered intestinal epithelial homeostasis in mice with intestine-specific deletion of the Krüppel-like factor 4 gene. *Developmental Biology*.

[24] Norman B., Davis J., Piatigorsky J. (2004). Postnatal gene expression in the normal mouse cornea by SAGE. *Investigative Opthalmology & Visual Science*.

[25] Segre J. A., Bauer C., Fuchs E. (1999). Klf4 is a transcription factor required for establishing the barrier function of the skin. *Nature Genetics*.

[26] Garrett-Sinha L. A., Eberspaecher H., Seldin M. F., de Crombrugghe B. (1996). A gene for a novel zinc-finger protein expressed in differentiated epithelial cells and transiently in certain mesenchymal cells. *Journal of Biological Chemistry*.

[27] Behr R., Kaestner K. H. (2002). Developmental and cell type-specific expression of the zinc finger transcription factor Krüppel-like factor 4 (Klf4) in postnatal mouse testis. *Mechanisms of Development*.

[28] Wen Y., Lu X., Ren J. (2019). KLF4 in macrophages attenuates tnf*α*-mediated kidney injury and fibrosis. *Journal of the American Society of Nephrology*.

[29] Wei D., Gong W., Kanai M. (2005). Drastic down-regulation of Krü Ppel-like factor 4 expression is critical in human gastric cancer development and progression. *Cancer Res*.

[30] Palumbo A., Anderson K. (2011). Multiple myeloma. *New England Journal of Medicine*.

[31] Pawlyn C., Davies F. E. (2019). Toward personalized treatment in multiple myeloma based on molecular characteristics. *Blood*.

[32] Kyle R. A., Rajkumar S. V. (2008). Multiple myeloma. *Blood*.

[33] García-Ledo L., Nuevo-Tapioles C., Cuevas-Martín C. (2017). Overexpression of the ATPase inhibitory factor 1 favors a non-metastatic phenotype in breast cancer. *Frontiers Oncology*.

[34] Allegra A., Innao V., Polito F., Oteri R., Aguennouz M. (2021). SIRT2 and SIRT3 Expression Correlates with Redox Imbalance and Advanced Clinical Stage in Patients with Multiple Myeloma. *Clinical Biochemistry*.

[35] Ding T., Hao J. (2021). Sirtuin 2 knockdown inhibits cell proliferation and RAS/ERK signaling, and promotes cell apoptosis and cell cycle arrest in multiple myeloma. *Molecular Medicine Reports*.

[36] Cui J., Shi M., Quan M., Xie K., Min S., Cui J. (2013). Regulation of EMT by KLF4 in gastrointestinal cancer. *Current Cancer Drug Targets*.

[37] Yori J. L., Johnson E., Zhou G., Jain M. K., Keri R. A. (2010). Krüppel-like factor 4 inhibits epithelial-to-mesenchymal transition through regulation of E-cadherin gene expression. *Journal of Biological Chemistry*.

RETRACTED

[38] Liu Y. N., Abou-Kheir W., Yin J. J. (2019). *Critical and Reciprocal Regulation of Klf4 and Slug in Transforming Growth Factor -initiated Prostate Cancer Epithelial-Mesenchymal Transition*.

[39] Leon S. P., Folkerth R. D., Black P. M. (1996). Microvessel density is a prognostic indicator for patients with astroglial brain tumors. *Cancer*.

[40] Chen H.-F., Wu K.-J. (2016). Endothelial transdifferentiation of tumor cells triggered by the twist1-jagged1-KLF4 Axis: relationship between cancer stemness and angiogenesis. *Stem Cells International*.

